# A New Measure of Pulse Rate Variability and Detection of Atrial Fibrillation Based on Improved Time Synchronous Averaging

**DOI:** 10.1155/2021/5597559

**Published:** 2021-04-01

**Authors:** Xiaodong Ding, Yiqin Wang, Yiming Hao, Yi Lv, Rui Chen, Haixia Yan

**Affiliations:** Shanghai Key Laboratory of Health Identification and Assessment, Laboratory of Traditional Chinese Medicine Four Diagnostic Information, Shanghai University of Traditional Chinese Medicine, Shanghai, China

## Abstract

**Background:**

Pulse rate variability monitoring and atrial fibrillation detection algorithms have been widely used in wearable devices, but the accuracies of these algorithms are restricted by the signal quality of pulse wave. Time synchronous averaging is a powerful noise reduction method for periodic and approximately periodic signals. It is usually used to extract single-period pulse waveforms, but has nothing to do with pulse rate variability monitoring and atrial fibrillation detection traditionally. If this method is improved properly, it may provide a new way to measure pulse rate variability and to detect atrial fibrillation, which may have some potential advantages under the condition of poor signal quality.

**Objective:**

The objective of this paper was to develop a new measure of pulse rate variability by improving existing time synchronous averaging and to detect atrial fibrillation by the new measure of pulse rate variability.

**Methods:**

During time synchronous averaging, two adjacent periods were regarded as the basic unit to calculate the average signal, and the difference between waveforms of the two adjacent periods was the new measure of pulse rate variability. 3 types of distance measures (Euclidean distance, Manhattan distance, and cosine distance) were tested to measure this difference on a simulated training set with a capacity of 1000. The distance measure, which can accurately distinguish regular pulse rate and irregular pulse rate, was used to detect atrial fibrillation on the testing set with a capacity of 62 (11 with atrial fibrillation, 8 with premature contraction, and 43 with sinus rhythm). The receiver operating characteristic curve was used to evaluate the performance of the indexes.

**Results:**

The Euclidean distance between waveforms of the two adjacent periods performs best on the training set. On the testing set, the Euclidean distance in atrial fibrillation group is significantly higher than that of the other two groups. The area under receiver operating characteristic curve to identify atrial fibrillation was 0.998. With the threshold of 2.1, the accuracy, sensitivity, and specificity were 98.39%, 100%, and 98.04%, respectively. This new index can detect atrial fibrillation from pulse wave signal.

**Conclusion:**

This algorithm not only provides a new perspective to detect AF but also accomplishes the monitoring of PRV and the extraction of single-period pulse wave through the same technical route, which may promote the popularization and application of pulse wave.

## 1. Introduction

The radial artery pulse wave is an important signal in health monitoring and disease diagnosis, which contains abundant physiological information. Different from the ECG signal which is often used to detect all kinds of arrhythmias [1], the radial artery pulse wave not only contains the information of heart rate and its variability which is widely used in smart watches and other wearable devices [2–4] but also can assist conventional methods to diagnose and monitor the occurrence and development of multiple common diseases such as hypertension, diabetes, and coronary heart disease [5–10]. In addition, the acquisition of radial artery pulse wave is much more convenient than ECG. However, except for atrial fibrillation (AF) detection and other the applications closely related to pulse rate variability (PRV), most of the applications depend on the information contained in single-period pulse waves. Due to the susceptibility of wearable devices to interference, it is so difficult to collect valuable single-period pulse waves with existing wearable devices that the information contained in the single-period pulse waves is neglected by wearable device researchers. Even for PRV monitoring and AF detection algorithms, it is imperative that subjects remain stationary during pulse wave acquisition. The application of pulse wave is restricted by the weak anti-interference ability.

Time synchronous averaging (TSA) is a widely used signal processing technique which enables periodic waveforms to be extracted from noisy signals [11, 12]. It is traditionally suited for the vibration analysis of mechanical systems which move circularly such as gearboxes. The noise of such signals can be effectively averaged out by gradually accumulating those portions of the signals that are synchronized with the fiducial points. Different from other noise reduction methods, TSA can effectively reduce all independent noise without considering frequency properties and threshold selection. Moreover, the signal-period pulse wave quality evaluation method [13] can be incorporated in TSA to identify and eliminate the seriously interfered periods. That is to say, we can select the less interfered periods from a pulse wave series with poor quality to complete TSA, rather than discarding the whole series (Figure 1). Similar algorithms have been applied to single-period pulse waveform extraction [14, 15]. However, in existing applications, the pulse wave signal is assumed to be a strict periodic signal, and the starting point or the highest point of the waveform is used as the fiducial point for synchronization without discussing the basis of these steps. More importantly, the single-period pulse wave extracted by existing TSA method does not contain the PRV information. It has nothing to do with PRV monitoring and AF detection. This may be the reason why TSA is neglected by wearable device researchers.

However, if we take two adjacent periods as the basic unit to calculate the average signal, it can be expected that with the increasement of PRV, the waveform of the second period will be gradually distorted due to the misalignment (Figure 2). The difference between waveforms of the two adjacent periods obtained by TSA may provide a new measure of PRV. Compared with traditional PRV measures, it may have some potential advantages under the condition of poor signal quality. And this index mainly reflects the irregular changes of heart rate. For patients with premature contraction (PC) which usually have regular changes in heart rhythm, the difference between adjacent periods may not be large because there are still a considerable number of second period waveforms are synchronous. The new index may effectively distinguish AF from PC and sinus rhythm (SR).

The objective of this paper was to develop a new measure of PRV by improving existing TSA and to detect atrial fibrillation by the new measure of pulse rate variability.

## 2. Methods

### 2.1. Data

In this study, the radial artery pulse wave signals were taken from 112 inpatients who had underwent an electrocardiographic (ECG) examination at Shanghai Shuguang Hospital between July 2019 and January 2020, including 11 cases with AF, 8 cases with PC, and 93 cases with SR. For each subject, a left radial artery pulse wave signal with a length of 60 seconds was taken by a wrist-type pulse wave monitor (type: Smart TCM-I, product by: Shanghai Asia & Pacific Computer Information System CO, Ltd, Shanghai, China) after the subject was either sitting or lying down for at least 5 min. ECG examination and pulse wave acquisition were performed on the same day but not simultaneously.

### 2.2. Preprocessing

The steps of preprocessing, including period segmentation and signal quality evaluation, are illustrated in Figure 3.

To segment the pulse wave series into periods, the derivative of the original signal was used to locate segmentation points by the threshold method (Figure 4). During threshold determination, each pulse wave series was segmented with 9 trial thresholds (0.1, 0.2, 0.3, 0.4, 0.5, 0.6, 0.7, 0.8, and 0.9). All the obtained segments were evaluated by a logistic regression model [13] which can divide the segments into normal segments and abnormal segments. The threshold with which the maximum number of normal segments were obtained was selected for the next steps.

During signal quality evaluation, the segment obtained by period segmentation were divided into normal and abnormal segments by the same logistic regression model as used in threshold determination. The abnormal segments were eliminated, and the range of normal segment was expanded by 50% on both sides to prepare for the measurement of PRV (Figure 5).

### 2.3. Time Synchronous Averaging

How to average the single-period pulse waves with different lengths in the same sequence and what is the appropriate fiducial point with the strongest anti-interference ability are questions that have not been fully discussed in current applications of TSA.

As shown in Figure 2, even in the pulse wave of a patient with AF, all the systoles have similar lengths and shapes, and the difference of cardiac cycle duration is mainly caused by the difference of diastolic duration. It is because the process of myocardial contraction and the state of arterial vessels are relatively stable for the same individual, and the duration of diastole does not significantly affect the left ventricular end-diastolic volume due to the low rate of left ventricular filling during late diastole. The initial condition and process of systole are basically stable. It is an appropriate averaging method to accumulate and average the preprocessed data without any stretching or compression, because most of the common time-domain features except the duration of cardiac cycle and diastole are extracted from the pulse wave of systole.

Figure 4 shows a pulse wave series and its derivative. The derivative of the original signal is almost entirely unaffected by baseline wander and shows clearer segmentation points. The spikes of the derivative are formed by the periodic rapid ejections of blood from the left ventricle. Different from the starting point or the highest point of a period where the waveform is relatively gentle and easy to be distorted by external interference, the spikes of the derivative have stronger anti-interference ability because the change of pulse wave caused by rapid ejection of blood is more significant than that caused by external interference. Moreover, the QRS complex, which is the most frequently used heartbeat fiducial point to calculate the heart rate in ECG [16], is formed by the same cardiac event. Using the peak of the derivative in each period as the reference point, the calculated results may have better comparability with the results of ECG. Therefore, the peak of the derivative is an appropriate fiducial point for synchronization of TSA.

Therefore, during TSA, the expanded single-period pulse waveforms obtained by preprocessing were synchronized with the maximum derivative value of each period, and all the waveforms from one pulse wave series were averaged directly without stretching or compression. After synchronizing, all the expanded single-period pulse waveforms were unified to the same length by filling with 0. If *X*_*i*_ = {*x*_1_, *x*_2_, ⋯, *x*_*n*_} was an expanded single-period pulse waveform and *N* was the number of normal segments in the sequence, the average expanded single-period pulse waveform of the sequence was given by

(1) $$\begin{array}{c} X_{a}=\frac{1}{N}\overset{N}{\underset{i=1}{\sum }}X_{i}. \end{array}$$

### 2.4. Measure of PRV and Detection of AF

To find an effective index of PRV, 50 cases with SR were randomly selected from the data set to generate the simulated training set with a capacity of 1000. The testing set consisting of the other 62 cases (AF:11, PC:8, SR:43) was used to test the ability of the selected index to detect AF. The training set was generated according to a simple and commonly used identification criterion for irregular heart rhythm—there is a variation of more than 0.16 seconds between the longest cardiac cycle duration and the shortest cardiac cycle duration [17]. The detailed steps to generate the simulated training set are as follows (Figure 6):

1. 50 single-period pulse waveforms were extracted from pulse wave signals of the 50 selected cases by TSA
2. Considering that the cardiac cycle duration is usually between 0.6 s and 1 s, for each single-period pulse waveform, 20 random numbers (denoted by *T*_*b*_) which obey the uniform distribution *U* (0.6,1) were generated to simulate different cardiac cycle durations of different individuals. A total of 1000 base cardiac cycle durations were generated for the 1000 expected training samples
3. 1000 single-period pulse waveforms were generated by stretching or compressing the original single-period pulse waveform to make its length equal to *T*_*b*_. All the 1000 single-period pulse waveforms were randomly divided into arrhythmia group and control group with 500 waveforms in each group
4. Each training sample consists of 60 cardiac cycles, and the duration of each cardiac cycle fluctuates around the base duration *T*_*b*_. The duration of each cardiac cycle is given by *T* = *T*_*b*_ + Δ*T*. In arrhythmia group, Δ*T* obeys the uniform distribution *U* (-0.09, 0.09). Whereas in control group, Δ*T* obeys the uniform distribution *U* (-0.07, 0.07). A sequence of 60 durations was generated for each training sample. In arrhythmia group, the variation between the maximum value and the minimum value of 60 durations is less than 0.18 but usually more than 0.16. Whereas in control group, the variation between the maximum value and the minimum value of 60 durations is less than 0.14. It is in accordance with the identification criterion for irregular heart rhythm
5. 60 single-period pulse waveforms were generated by stretching or compressing the corresponding single-period pulse waveform generated in step 3 to make its length equal to the 60 durations separately. The pulse wave series of each training sample were subsequently obtained by connecting the 60 single-period pulse waveforms end to end. Considering that the systolic duration of an individual is almost constant, only the waveforms of diastole were stretched or compressed to satisfy the requirement of cardiac cycle durations in this step

After the training set was generated, the average expanded single-period pulse waveform of each training sample was extracted by TSA. The difference between the first ascending limb and the second ascending limb were tested to distinguish between arrhythmia group and control group. The first ascending limb is defined as the data between the minimum value and the maximum value in the first half of the expanded single-period pulse waveform. The second ascending limb is defined as the data starting from the minimum value between the maximum values of the first half and the second half of the expanded single-period pulse waveform and with the same length as the first ascending limb (Figure 7). Considering that Euclidean distance (*D*_e_), Manhattan distance (*D*_m_), and cosine distance (*D*_c_) are commonly used distance measures between two vectors, these 3 candidate indexes were tested on the training set to distinguish between arrhythmia group and control group. If *X*_*f*_ = {*x*_*f*1_, *x*_*f*2_, ⋯, *x*_*fn*_} and *X*_*s*_ = {*x*_*s*1_, *x*_*s*2_, ⋯, *x*_*sn*_} were the data of first ascending limb and the second ascending limb, respectively, *D*_e_, *D*_m_, and *D*_c_ were given by

(2) $$\begin{array}{c} D_{\text{e}}=\sqrt{\overset{n}{\underset{i=1}{\sum }}{\left(x_{fi}-x_{si}\right)}^{2}},\\ D_{\text{m}}=\overset{n}{\underset{i=1}{\sum }}\left|x_{fi}-x_{si}\right|,\\ D_{\text{c}}=\frac{\sum_{i=1}^{n}x_{fi}x_{si}}{\sqrt{\sum_{i=1}^{n}{x_{fi}}^{2}}\sqrt{\sum_{i=1}^{n}{x_{si}}^{2}}}. \end{array}$$

The receiver operating characteristic (ROC) curve was used to evaluate the performance of the indexes. The index with the maximum area under ROC curve (AUC) was selected to detect AF on the testing set. The distribution of the selected index in different groups of the testing set was compared by Kruskal-Wallis test. And the AF identification performance on the testing set was evaluated by ROC curve.

## 3. Results

### 3.1. Performance of Candidate Indexes on Training Set

The ROC curves of 3 candidate indexes on the training set are shown in Figure 8. The AUC of *D*_e_, *D*_m_, and *D*_c_ were 0.857, 0.801, and 0.516, respectively. Both *D*_e_ and *D*_m_ can effectively identify irregular pulse rhythm, and *D*_e_ performed best in this task.

### 3.2. Comparison of *D*_e_ in Different Groups of Testing Set

The comparison result of *D*_e_ in different groups of testing set by Kruskal-Wallis test is shown in Table 1. And the box-plot of *D*_e_ in different groups of testing set is shown in Figure 9. The result indicated that *D*_e_ in AF group is significantly higher than that of the other two groups, and there was no significant difference between the PC and SN group. Therefore, *D*_e_ can be used as an indicator to detect AF.

### 3.3. Performance of *D*_e_ to Detect AF on Testing Set

The ROC curve of *D*_e_ to identify AF on the testing set are shown in Figure 10. The AUC was 0.998, and the accuracy, sensitivity, and specificity were 98.39%, 100%, and 98.04%, respectively, with the threshold of 2.1. *D*_e_ can effectively detect AF from pulse wave signals.

### 3.4. Comparison with Other Works

With the popularity of wearable devices, the research of AF detection based on pulse wave is increasing in recent years (Table 2). However, except Shannon entropy, most of the features used to detect AF are based on the interbeat interval (IBI) series, which makes the accurate calculation of the cardiac cycle duration a prerequisite for AF detection. Therefore, the sensitivity to external interference has become a common weakness of these studies. As indicated in Table 2, the method proposed in this paper is one of the most accurate methods. And it does not rely on IBI series, consequently, and may have stronger anti-interference ability.

## 4. Discussion

In this paper, we propose a new measure of PRV based on TSA. It was discovered that this new index can effectively detect AF from pulse wave signals. It can not only be applied to the seriously interfered signal by combining with single-period pulse wave quality evaluation method, but also extract a high-quality single-period pulse waveform at the same time, which can be used in other pulse wave-related applications. In addition, it can distinguish AF and PC, which has long been a problem in the identification of AF [21].

Figure 11 shows a typical average pulse wave of PC. Although the PRV of patient with PC is large, the change of its cardiac cycle durations is usually regular. Therefore, there are still enough synchronized second ascending limbs to form a similar average waveform with the first ascending limbs. The other second ascending limbs will form the bulge in the red box of Figure 9. This feature is usually located in the diastolic of the average waveform. The diastolic pulse wave of healthy people usually decreases gradually without obvious features. This feature may be used to detect PC in the future.

In summary, the new index provides a new perspective to measure PRV and to detect AF. Moreover, it accomplishes the monitoring of PRV and the extraction of single-period pulse wave through the same technical route, which may promote the popularization and application of pulse wave. However, this study also has limitations: (1) the sample size is so limited that we had to use simulated data instead of real clinical data to screening candidate indexes. Therefore, *D*_e_ may not be the best choice for real clinical data. (2) The ECG and pulse wave are not collected simultaneously, which may lead to incorrect label. (3) The anti-interference ability has not been verified because the new index was not tested on seriously interfered data set.

In the future, we hope to improve this algorithm by collecting more real clinical data and screening more distance measures. In addition, it has been discovered that there is a unique characteristic on the average pulse wave of PC. It is also one of the future research directions to develop an automatic PC detection algorithm based on this characteristic.

## Figures and Tables

**Figure 1:** General steps of TSA combined with signal-period pulse wave quality evaluation method. (a) A pulse wave series was segmented into periods. (b) The signal quality of each segment was evaluated, and the abnormal segments were eliminated. (c) All the normal segments were synchronized with the starting points. (d) The noise was suppressed by averaging the synchronized signals.

**Figure 2:** The average pulse wave with a basic unit of two adjacent periods. (a) The average pulse wave of a normal individual. The waveforms of the two adjacent periods are similar. (b) The average pulse wave of a patient with AF. The waveform of the second period is seriously distorted.

**Figure 3:** Steps of preprocessing. During period segmentation, the original pulse wave series were segmented into periods by threshold method. During signal quality evaluation, the segment obtained by period segmentation were divided into normal and abnormal segments by a logistic regression model. The abnormal segments were eliminated, and the range of normal segment was expanded by 50% on both sides to include the information of adjacent periods.

**Figure 4:** Pulse wave and its derivative with an applied threshold. The derivative of the original signal is almost entirely unaffected by baseline wander and shows clearer segmentation points. The first zero point of the derivative before each threshold point was defined as the period segmentation point, and the corresponding segments of the original signal between two adjacent period segmentation points were single-period waveforms.

**Figure 5:** Expanded single-period pulse wave. The range of each segment was expanded by 50% on both sides to include the information of adjacent periods.

**Figure 6:** Steps to generate the simulated training set. (a) 50 single-period pulse waveforms were extracted from pulse wave signals of the 50 selected cases by TSA. (b) 1000 single-period pulse waveforms were generated by stretching or compressing the original single-period pulse waveform to make its length equal to *T*_*b*_. (c) 60 single-period pulse waveforms were generated by stretching or compressing the corresponding single-period pulse waveform generated in (b) to make its length equal to *T*_*b*_ + Δ*T* separately. Only the waveforms of diastole were stretched or compressed in this step. The pulse wave series of each training sample were subsequently obtained by connecting the 60 single-period pulse waveforms end to end.

**Figure 7:** The first ascending limb and the second ascending limb of expanded single-period pulse wave. (a) The first ascending limb is defined as the data between the minimum value and the maximum value in the first half of the expanded single-period pulse waveform. (b) The second ascending limb is defined as the data starting from the minimum value between the maximum values of the first half and the second half of the expanded single-period pulse waveform and with the same length as the first ascending limb.

**Figure 8:** ROC curves of 3 candidate indexes on the training set. The AUC of *D*_e_, *D*_m_, and *D*_c_ are 0.857, 0.801, and 0.516, respectively.

**Figure 9:** Box-plot of *D*_e_ in different groups of testing set.

**Figure 10:** ROC curve of *D*_e_ to detect AF on the testing set. The AUC was 0.998, and the accuracy, sensitivity, and specificity were 98.39%, 100%, and 98.04%, respectively, with the threshold of 2.1.

**Figure 11:** A typical average pulse wave of PC. There are still enough synchronized second ascending limbs in pulse wave of PC to form a similar average waveform with the first ascending limbs. The other second ascending limbs will form the bulge in the red box.

**Table 1:** Comparison of *D*_e_ in different groups of testing set by Kruskal-Wallis test.

Groups	Test statistic	Standard error	*p*
SN-AF	32.049	6.096	<0.001
PC-AF	24.659	8.383	0.010
SN-PC	7.390	6.947	0.862

**Table 2:** Comparison of recent pulse-wave-based AF detection techniques.

Reference	Methods	Accuracy (%)
McManus DD, et al. (2013) [18]	RMSSD and Shannon entropy	96.76
Krivoshei L, et al. (2017) [19]	Shannon entropy and other IBI features	87.5
Fallet S, et al. (2019) [20]	Bagging decision tree based on IBI features	88.5
Kabutoya T, et al. (2019) [3]	Irregular heartbeat ratio	98.3
Kashiwa A, et al. (2019) [21]	IBI features	97.3
Zalabarria U, et al. (2020) [22]	ANN with foot point detection	93.68
Han D, et al. (2020) [23]	Random forest with Poincare plot	95.32
This paper	D_e_ between adjacent periods based on TSA	98.4

## Data Availability

The original data used to support the findings of this study are available at https://github.com/Xiaodong-Ding/AFDetect.

## Abbreviations

PRV: Pulse rate variability
AF: Atrial fibrillation
TSA: Time synchronous averaging
PC: Premature contraction
SN: Sinus rhythm
ROC: Receiver operating characteristic
AUC: Area under curve
ECG: Electrocardiographic
IBI: Interbeat interval.
